# Reconstruction of bone defect with autograft fibula and retained part of tibia after marginal resection of periosteal osteosarcoma: a case report

**DOI:** 10.1186/s12957-015-0618-2

**Published:** 2015-06-18

**Authors:** Tongyu Hu, Wei Chen, Jianheng Li, Chenguang Du, Yingze Zhang

**Affiliations:** Department of Orthopaedic Surgery, The Third Hospital of Hebei Medical University, Shijiazhuang, Hebei 050051 People’s Republic of China; Department of Orthopedic Surgery, Chinese People’s Liberation Army No. 256 Hospital, Shijiazhuang, Hebei 050041 People’s Republic of China

**Keywords:** Periosteal osteosarcoma, Marginal resection, Autograft fibula, Retained tibia, Chemotherapy

## Abstract

Periosteal osteosarcoma is a rare subtype of osteosarcoma. Wide surgical removal is the commonly used treatment-method algorithm. However, the limb-salvage procedure of periosteal osteosarcoma in the distal tibia is a technical challenge to orthopedic surgeons because of the scarcity of soft tissue and subcutaneous nature in the anteromedial aspect. We encountered a 16-year-old female patient with periosteal osteosarcoma in the distal half of the left tibia diagnosed preoperatively based upon the CT images and a needle biopsy. A unique identical surgical technique was applied in the case, including marginal resection of the periosteal osteosarcoma with part of the tibia retained at the same level of bone defect and reconstruction using the autologous fibula graft. A combination of cisplatin and doxorubicin was received as chemotherapy after the operation. Postoperative incisional biopsy was performed, and the hematoxylin-eosin-stained results confirmed the diagnosis of periosteal osteosarcoma. The patient was followed up for 11 years. Radiological and clinical evaluation was performed at each follow-up. The retained tibia incorporated well with the fibula autograft, and excellent limb functional recovery was achieved. The patient was free from neoplastic disease at the latest follow-up. In conclusion, young patients with periosteal osteosarcoma without intramedullary involvement can be treated by marginal resection of the lesion with part of the tibia retained at the level of bone defect and reconstructed using a long autologous fibula graft. Subsequent chemotherapy with administration of cisplatin and doxorubicin is recommended.

## Background

Periosteal osteosarcoma is a relatively well-differentiated chondroblastic osteosarcoma and is less aggressive than conventional osteosarcoma [1]. It often occurs on the surface of the long bones of the extremities [2]. The lesion locates most frequently on the diaphysis of the tibia and femur [3]. Wide surgical resection is the mainstay of treatment methods of periosteal osteosarcoma, which often leads to large diaphyseal bone defect [4]. The reconstruction of a large bone defect of the tibia is a surgical challenge because of the scarcity of soft tissue and the subcutaneous nature in the anteromedial aspect. There are no autologous bone grafts with proper size to bridge the gap in some cases with a large bone defect. In such a condition, we treat the lesions by marginal resection of the periosteal osteosarcoma with part of the tibia retained at the same level of bone defect and reconstruction using the autologous fibula graft harvested from the right lower extremity. The graft fibula and the retained tibia serve as the structure supporter. Here, we present such a case free from neoplastic disease recurrence at a follow-up period of 11 years.

## Case presentation

A 16-year-old girl presented with a 6-month history of intermittent pain and swelling over the anterior medial aspect of the distal diaphysis of her left tibia. The pain was exacerbated by activity and released by rest. The bony mass grew into 3 × 6 cm in size when she was administrated into our hospital. A palpable, immobile, and mild tender mass was noted 5 months prior to administration. The local skin appeared normal without redness and venous engorgement. The radiographs of the distal tibia shaft demonstrated a mass on the bone surface, which contained radiolucent and sclerotic regions. The radiographs also showed thickened underlying diaphyseal cortex and perpendicular periosteal reaction extending into the soft tissue mass (Fig. 1). Computed tomography was taken, and the lesion was about one half of the circumference of the tibia in width without obvious medullary involvement (Fig. 2). According to the radiological features, parosteal and periosteal osteosarcoma were considered. A needle biopsy was carried out. The hematoxylin-eosin-stained results revealed the lobules of neoplastic cartilage with myxoid matrix, which implied periosteal osteosarcoma.

**Fig. 1:** The radiographs demonstrate thickened diaphyseal cortex and perpendicular periosteal reaction extending into the soft tissue in the anteromedial aspect of the tibia. **a** Anteroposterior view; **b** lateral view

**Fig. 2:** Computed tomography reveals cortical thickening and extrinsic scalloping of the cortex without medullary involvement. **a** Axial image; **b** sagittal image

Marginal resection of the periosteal osteosarcoma was performed. At the time of surgery, the lesion margin was firstly identified based upon the CT findings. The lesion was approached by way of an anteromedial incision. Meticulous dissection was performed to preserve sufficient protective margins of tissue. The tumor was exposed and appeared as thickened and enlarged sclerotic bone without adjacent soft tissue mass. Surgical margin of the tumor was finally defined according to the CT images and gross inspection. The bone was excised more than 2 cm away from the margins of the tumor. The lesion and surrounding normal bone were removed. The bone block, about three fifths of the circumference in width and 12 cm in length of the affected tibia, was excised. A large bone defect was left. The retained tibia was about two fifths of the circumference in width at the level of bone defect, which maintained the nature continuity with that superior and inferior to the bone defect. Preliminary evaluation of the surgical margin and intramedullary cavity was performed immediately after removal of the tumor. The bony resection margins were judged clear, and the intramedullary aspect of the lesion was assessed to be uninvolved by gross observation.

A fibular autograft was harvested from the right lower leg to reconstruct the bone defect of the left tibia. A straight incision about 18 cm in length was made from the point 10 cm above the lateral malleolus along the posterior border of the fibula. The fibula was reached via the posterolateral approach. An 18-cm long fibular bone block was resected. Both ends of the fibular graft were trimmed, and the medullary canal of the tibia was reamed. The fibular graft was firmly impacted into the proximal and distal medullary canal of the left tibia. The wound was closed in order, and a plaster cast was applied to stabilize the calf, the knee, and ankle joints.

Incisional biopsy tissues were gained postoperatively from multiple sites of the resected tumor and along the surgical margins for histopathological analysis. The hematoxylin-eosin-stained results confirmed the preoperative diagnosis of periosteal osteosarcoma (Fig. 3), grade 2 according to the staging system of Enneking [5]. The histopathological examination showed that the margin of the specimen was clear from tumor cells, and no medullary involvement was identified. Postoperative radiographs of the left lower leg were taken, which demonstrate the retained tibia and the bone defect reconstructed with fibular autograft and stabilized using a plaster cast (Fig. 4). The patient received chemotherapy, a combination of cisplatin and doxorubicin, as would be used for conventional osteosarcoma [6–8].

**Fig. 3:** Low-power view reveals typical periosteal osteosarcoma features, which consisted of the lobules of neoplastic cartilage and myxoid matrix, surrounded by fibrous membrane; the cartilage composed of atypical chondroblastic cells (hematoxylin and eosin, ×40)

**Fig. 4:** The radiographs demonstrate the retained tibia and fibula graft in the bone defect. **a** Anteroposterior view; **b** lateral view

The postoperative course was uneventful. The patient was encouraged to perform isometric muscle exercises of the affected lower extremity and full range of motion of the hip joint as soon as pain could be tolerated. Non-weight-bearing crutch walking was allowed after soft tissue healing. The cast was removed at 3 months postoperatively, and partial weight bearing was permitted, progressing to full weight bearing at 6 months. Follow-up was conducted at 1, 3, 6, and 12 months after the operation and every year thereafter. Radiological and clinical evaluation was performed at each follow-up. Excellent bony healing of the tibia and fibula graft was observed on the radiographs of the left lower limb at 6 months, and the patient regained normal walking function without a crutch. The retained tibia at the bone defect level grew and gradually wrapped the fibula graft. The tibia incorporated well with the fibula graft at 36 months postoperatively. The radiographs at 60 months of follow-up demonstrated that the fibula graft was almost absorbed. The reconstructed tibia nearly regained the diameter as the contralateral unaffected tibia (Fig. 5). At the latest follow-up, 11 years after the operation, the radiographs and CT scan of the bilateral lower extremities were taken, showing good remolding of the retained tibia and fibular autograft (Figs. 6 and 7). The muscle strength of the bilateral lower limbs were evaluated both as normal (grade 5) according to the Manual Muscle Testing Grading System. Single-legged hop tests [9, 10] were conducted, and the patient was classified as having self-reported normal function of the bilateral knees. The patient can now conduct daily activities and manual work with a score of 100 according to the Activities of Daily Living (ADL) questionnaire. During the follow-up period of 11 years after surgery, no local recurrence or distant metastasis occurred in the patient.

**Fig. 5:** **a**, **b** The radiographs show that the fibula graft is almost absorbed, and the tibia is nearly as thick as the contralateral tibia at 60-month follow-up

**Fig. 6:** At the 11-year follow-up, the radiographs of the bilateral lower extremities demonstrated good remolding of the retained tibia and fibular autograft. **a** Anteroposterior view of *right* tibia, **b** lateral view of *right* tibia, **c** anteroposterior view of the *left* tibia, and **d** lateral view of the *left* tibia

**Fig. 7:** Computed tomography taken at the latest follow-up reveals good remolding of the retained tibia and fibular autograft. **a** Coronal view, **b** sagittal view, and **c** 3-D reconstruction

### Discussion

In the current study, we treated a young female patient with periosteal osteosarcoma by marginal resection with retained tibia at the same level of bone defect and reconstruction using the autologous fibula graft. Chemotherapy was received postoperatively. The retained tibia incorporated with the graft fibula well, and excellent limb function was achieved. Local recurrence or distal metastasis was not reported at the 11-year follow-up.

Periosteal osteosarcoma was described in 1976 by Unni and his colleagues [11]. Histologically, it consists of a large chondroblastic tissue with smaller areas of osteoid formation [3]. Radiographically, it appears as a well-defined, essentially radiolucent mass probably with cortical thickening, extrinsic scalloping of the cortex, and periosteal reaction. CT and magnetic resonance (MR) imaging can reveal the extent of the soft tissue mass. The large chondroid tissue is demonstrated as low attenuation at CT and high signal intensity at T2-weighted MR imaging. There is only occasional involvement of the underlying cortex. The involvement of the medullary cavity is significantly rare. Pathologically, periosteal osteosarcoma is an intermediate-grade chondroblastic osteosarcoma (grade 2 or 3) [12–15].

Surgery is required to cue periosteal osteosarcoma, and wide surgical excision is regarded as an appropriate therapy [11, 13, 16]. However, a large bone defect is often a leftover after wide resection. There are no autologous bone grafts with proper size to bridge the gap in such cases. Massive allografts are prone to infection [17]. Alternatively, marginal section is also an option taking the low malignance of periosteal osteosarcoma into consideration. Since local recurrence has a tendency to occur in case of incomplete resection, the bony resection margins and the intramedullary aspect of the lesion should be confirmed as clear at the time of surgery.

Periosteal osteosarcoma occurs most often in adolescents and has a predilection for the diaphysis of the tibia or the femur [16]. The young patients have high demand of the limb function. Limb-salvage surgery should be performed in these patients. The limb-salvage procedure of a malignant tumor in the distal tibia is a great challenge to orthopedic surgeons. The distal half of the diaphysis of the tibia has a few direct muscle attachments, and only part of posterior tibialis posterior, flexor digitorum longus, and extensor digitorum longus are originated from the distal half of the tibia. The limb salvage presents unique difficulties [18].

To reduce the difficulty encountered in the limb-salvage surgery and preserve the limb function to the utmost extent, we treat the periosteal osteosarcoma by marginal resection. The lesion and its surrounding normal bone was excised in the affected segment of the tibia. Part of the tibia at the same level of bone defect was retained to maintain the continuity of the cortex. The retained tibia served as the structure supporter of the lower limb and preserved the limb length. The bone defect was reconstructed with a long autograft fibula, which was trimmed and inserted into the intramedullary cavity. The fibula graft had the following two main functions: improving the osteogenesis and providing structure support. No implant was needed. Accordingly, implant-related complications or implant removal was avoided. The tibia incorporated well with the autograft fibula at 36 months after surgery as demonstrated on CT. The fibula graft was almost absorbed, and the reconstructed tibia was nearly as thick as the contralateral unaffected tibia. The muscle strength of the left lower extremities was evaluated according to the Manual Muscle Testing Grading System, and functional recovery of the left knee joint assessed using single-legged hop tests were both normal. The patient can now conduct daily activities and manual work without any difficulty. Compared with limb-salvage surgery using prosthesis, the novel technique is easy to perform. It is also economy-friendly, especially in the developing country.

At the latest follow-up, no local recurrence or distal metastasis was reported. Two factors may contribute to these issues. At the time of surgery, the bony resection margins and the intramedullary aspect of the lesion were judged clear. Postoperative histopathological examination confirmed the intraoperative judgment. In addition, the cisplatin and doxorubicin were applied in the case. Controversy remains as to whether chemotherapy is necessary in the management of periosteal osteosarcoma [1, 11, 19, 20]. Previous studies have produced mixed results in this consideration. In the report of Bertoni et al., a marginal excision was done in eight patients with periosteal osteosarcoma, and all but one was affected by a local recurrence [13]. Chemotherapy was not used in the initial treatment in their study. Grimer and his colleagues also reported that the use of chemotherapy was not shown to be a prognostic factor, but the chemotherapy was used in two thirds of the patients (80 patients) in their study, and doxorubicin and cisplatin were used in 75 patients (93.8 %) [21]. Revell and his colleagues claimed 100 % survival in patients who have undergone adequate chemotherapy and surgery [22]. While in our study, pre- and postoperative chemotherapy were used, and no recurrence was found during the follow-up period of 11 years.

Although the presented case demonstrated excellent functional recovery without local recurrence or distal metastasis for a long term of follow-up, this procedure should be restricted to low-grade periosteal osteosarcoma without medullary involvement. Larger numbers and a longer follow-up are needed to verify the efficacy of this kind of reconstruction fairly.

## Conclusions

This unique surgical technique, including marginal resection of periosteal osteosarcoma with part of the tibia retained at the same level of bone defect and reconstruction using autologous fibula graft, and postoperative chemotherapy, can be applied effectively in the treatment of young patients. The patient has been continuously disease-free during the follow-up period of 11 years after surgery. The muscle strength of the bilateral lower limbs were evaluated according to the Manual Muscle Testing Grading System, and the bilateral knee functions assessed using single-legged hop tests were both normal. This treatment algorithm at our institution shed light on the management of similar cases.

## Consent

The patient and her family were informed that the data of the case would be submitted for publication and gave their informed consent.

### Institutional review board statement

This material has not been published and is not under consideration elsewhere. There is no financial disclosure from each author.
